# The causal relationship between immune cells mediating FIT3L, CCL4, OSM, and skin‐derived deteriorated tumors

This article has been retracted.

**DOI:** 10.1111/srt.13774

**Published:** 2024-07-02

**Authors:** Wanli Gong, Jiayi Zhou, Yaqi Hou, juan Zhang, Peifeng He, Qi Yu

**Affiliations:** ^1^ School of Management Shanxi Medical University Jinzhong Shanxi China; ^2^ Key Laboratory of Big Data in Clinical Decision Research Shanxi Medical University Taiyuan Shanxi China; ^3^ Faculty of Arts and Social Sciences University of Sydney Broadway Australia

**Keywords:** basal cell carcinoma, circulating inflammatory proteins, cutaneous malignant melanoma, cutaneous squamous cell carcinoma, immune cells, two‐step Mendelian randomization

## Abstract

**Objective:**

Observational studies have identified a dual effect of circulating inflammatory proteins and immune cells on cancer progression. However, the specific mechanisms of action have not been clarified in the exacerbation of cutaneous‐origin tumors. Therefore, this study aims to investigate whether the causal relationship between circulating inflammatory factors and basal cell carcinoma (BCC), cutaneous malignant melanoma (SKCM), and cutaneous squamous cell carcinoma (cSCC) is regulated by immune cells.

**Methods:**

This study employed the Two‐Sample Mendelian Randomization (TSMR) approach to investigate the causal relationships between 91 circulating inflammatory factors and three prevalent types of skin cancer from a genetic perspective. Bayesian Weighted Mendelian Randomization (BWMR) was also used to validate correlation and reverse MR to assess inverse relationships. Subsequent sensitivity analyses were conducted to limit the impact of heterogeneity and pleiotropy. Finally, the two‐step Mendelian Randomization (two‐step MR) method was utilized to ascertain the mediating effects of specific immune cell traits in the causal pathways linking circulating inflammatory factors with BCC, SKCM, and cSCC.

**Results:**

The Inverse Variance Weighted (IVW) method and the Bayesian Weighted Algorithm collectively identified nine inflammatory factors causally associated with BCC, SKCM, and cSCC. The results from Cochran's Q test, mendelian randomization pleiotropy residual sum and outlier (MR‐PRESSO), and MR‐Egger intercept were not statistically significant (*p* < 0.05). Additionally, the proportions mediated by CD4+ CD8dim T cell %leukocyte, CD4‐CD8‐Natural Killer T %T cell, and CD20 on IgD‐CD38‐B cell for FIt3L, CCL4, and OSM were 9.26%, 8.96%, and 10.16%, respectively.

**Conclusion:**

Immune cell levels potentially play a role in the modulation process between circulating inflammatory proteins and cutaneous‐origin exacerbated tumors. This finding offers a new perspective for the in‐depth exploration of cutaneous malignancies.

## 1 INTRODUCTION

Cutaneous malignancies include Basal cell carcinoma (BCC), Skin cutaneous melanoma (SKCM), and Cutaneous squamous cell carcinoma (cSCC), among others. BCC, as the most common cutaneous malignancy globally, has an incidence rate of up to 4.3 million cases.^1^ It is predominantly treated with surgery and generally has a good prognosis. According to the european association of dermato‐oncology (EADO) classification, BCC is classified as easy to treat or difficult to treat.^2^ SKCM is more malignant, and factors such as pesticide use, sun exposure, and geographic location may increase its risk of incidence.^3^ Surgical excision is the mainstay treatment method for SKCM, while systemic drug therapy, as an adjunctive approach, has been proven to significantly improve survival rates in SKCM patients.^4^ cSCC is the second most common type of non‐melanoma skin cancer after BCC, and epidemiological studies indicate that its incidence is also on the rise.^5^ The AJCC‐8 tumor, node, and metastasis (TNM) staging system is applied to cSCC staging, where T1‐T2 are key features in determining the severity of the disease. The prognosis for advanced cSCC is generally poor.^6^ Therefore, exploring new targets and pathogenic mechanisms is particularly crucial for improving treatment outcomes. With the in‐depth study of the pro‐carcinogenic and anti‐carcinogenic functions of circulating inflammatory proteins, numerous opportunities are provided to achieve these goals.

Circulating inflammatory proteins are involved in the regulation of immune functions, signal transduction, and cell activation, playing a pivotal role in the body's immune defense and tumor development. Various cytokines actively regulate the occurrence and progression of tumors. The significant pro‐carcinogenic effects of IL‐6 (interleukin‐6), IL‐1β (interleukin‐1 beta), and TGF‐β (transforming growth factor beta) have been confirmed, involving cancers such as lung and breast cancer.^7^ In contrast, cytokines like IL‐2 (interleukin‐2) and IL‐12 (interleukin‐12) can positively regulate the tumor suppression process.^8^ Meanwhile, there are cytokines like TNF‐α (tumor necrosis factor‐alpha) that possess dual pro‐carcinogenic and anti‐carcinogenic roles. Cytokines and chemokines influence tumors directly or indirectly by regulating the migration, activation, and function of immune cells,^9^ revealing the mediating role of immune cells in the process of cytokine‐regulated tumors.

Immune responses are closely related to tumor development and prognosis. The immune system plays a crucial role in both the promotion and suppression of BCC.^10^ Immune checkpoint inhibitors have been widely used in various cancers, including BCC, SKCM, and Cscc.^4^ However, the extent to which immune cells regulate tumor development remains unclear. Mendelian randomization (MR) utilizes genetic variations associated with modifiable exposure factors to explore potential causal relationships between these variations and specific outcomes.^11^ As one of the most effective tools for assessing causality, it can minimize confounding factors and enhance the robustness of observational study results.

This study used recently acquired large‐scale public GWAS summary statistics and explored the mediating level of immune cells in the potential causal relationship between circulating verification proteins and cutaneous‐origin exacerbated tumors through Two‐Sample Mendelian Randomization (TSMR), inverse MR, Bayesian Weighted Mendelian Randomization (BWMR), and two‐step MR.

## 2 MATERIALS AND METHODS

### 2.1 Research design

In this study, single nucleotide polymorphisms (SNPs) are considered as IVs for exploring causality. Eligible instrumental variables (IVs) need to satisfy the following assumptions: genetic variations are independent of confounding factors, genetic variations are significantly associated with circulating inflammatory proteins, and there are no alternative pathways through which genetic variations affect cutaneous‐origin exacerbated tumors.^12^ On this basis, the causal effects between exposure factors and outcomes were further explored, including total, indirect, and direct effects (Figure 1). First, using large‐scale public genome‐wide association study (GWAS) summary data, the total causal effect of circulating inflammatory proteins and cutaneous‐origin exacerbated tumors is estimated through bidirectional, TSMR. Concurrently, BWMR further validates the causal relationship. Subsequently, the two‐step MR analysis strategy is used to assess the indirect causal effect mediated by immune cell traits. The direct effect is calculated via the method of coefficient differences. Finally, this causal analysis adheres throughout to the Strengthening the Reporting of Observational Studies in Epidemiology (STROBE) guidelines to ensure the scientific rigor and standardization of the study.^11^

**FIGURE 1:** Analytical Approach of TSMR and two‐step MR. MR, Mendelian Randomization; TSMR, Two‐Sample Mendelian Randomization.

### 2.2 Data acquisition

The GWAS summary statistics for the exposure factors were derived from a meta‐analysis involving 11 cohorts with a total of 14 824 European participants. This study utilized the Olink Target platform for the measurement of genomic genetic data and plasma proteome data, identifying a total of 91 circulating inflammatory proteins.^13^ The related complete data are accessible from the public open database GWAS Catalog (https://www.ebi.ac.uk/gwas/) with IDs ranging from GCST90274758 to GCST90274848.

A new GWAS involving 3757 individuals from Sardinia identified over 20 million SNPs and 731 genetic components associated with immune phenotypes, including 539 immune cell‐related traits and 192 relative counts.^14^ The OpenGWAS database (https://gwas.mrcieu.ac.uk/) provided the most comprehensive genetic statistics related to immune cells for this study. This dataset, published in 2020, is accessible with IDs ranging from GCST90001391 to GCST90002121.

The FinnGen database integrates genetic information, clinical data, and health records from over 400 000 Finnish individuals, aiming to provide robust support for unveiling disease mechanisms, drug development, and personalized medicine. The ninth version of this database supplied the outcome data for this study. Specifically, the BCC summary statistics incorporated data from 18 982 European ancestry patients and 287 137 control individuals. SKCM and cSCC included 2993 and 3251 European patients, respectively.

Given that the GWAS data for cutaneous‐origin exacerbated tumors, circulating inflammatory proteins, and immune cell‐related traits are all sourced from different publicly accessible platforms, the likelihood of sample overlap is minimized. Additionally, the selected datasets for this study have been publicly published, obviating the need for additional ethical review.

### 2.3 Instrumental variable selection

First, SNPs closely associated with circulating inflammatory proteins were identified using a threshold of *p* < 5 × 10^‐8^ to meet the relevance assumption. To incorporate a sufficient number of positive SNPs into the analysis, this study expands the selection criteria to 1 × 10^‐5^.^15^ Additionally, the clump data method from the R package Two‐Sample MR is employed to remove errors caused by linkage disequilibrium effects (*kb* = 10 000, *R* ^2^ = 0.001), ensuring the independence of SNPs. Subsequently, the harmonize_data() function is used to eliminate palindromic sequences, thereby ensuring higher reliability and accuracy of genetic markers. Next, SNP strength is assessed using the formula *F* = *β* ^2^/SE^2^, with an *F*‐value threshold of < 10 to exclude weak IVs.^16^ Finally, potential confounders for SNPs (such as albinism, obesity, and human papillomavirus) are filtered out via the LDlink website (https://ldlink.nih.gov/).

### 2.4 Analysis

MR analyses were conducted using the R packages Two‐Sample MR and MR. The IVW method was selected as the primary analysis approach. When IVs are not pleiotropic, IVW is the most efficient method with valid instruments and accounts for the heterogeneity of variant‐specific causal estimates.^17^ Meanwhile, MR‐Egger regression and the Weighted Median Estimator (WME) were used to reinforce causal inference, with BWMR used to verify causal relationships. The MR‐Egger method allows for pleiotropic effects in all genetic variants, thus providing causal estimates even when all IVs are invalid.^17^ BWMR enhances the robustness of causal inference by effectively removing interferences that violate the IV assumptions and corrects the posterior covariance, thereby strengthening the reliability of the causal effect.^18^

To facilitate the interpretation of causal relationships, the derived *β* values are converted into Odds Ratio (OR), with the corresponding 95% confidence intervals (CI) also calculated.

### 2.5 Sensitivity analysis

To verify the robustness of the causal relationship and eliminate key factors that might affect the causal assumptions, a series of quality control measures were implemented to assess the sensitivity, heterogeneity, and pleiotropy of the study outcomes. Initially, Cochran's Q test was employed via the IVW method to calculate its derived *p*‐value, aiming to eliminate the influence of heterogeneity. Subsequently, the MR‐PRESSO global test and MR‐Egger intercept were used to correct for horizontal pleiotropy after outlier exclusion. Lastly, a leave‐one‐out analysis was conducted, where the leave‐one‐out() function sequentially excluded each IV to reperform the causal analysis, comparing the extent to which the results were affected.

Additionally, this study applied the Bonferroni correction to mitigate the potential impact of multiple testing. A *p*‐value of < 0.0005 (0.05/91) was considered strong evidence. While results with *p*‐values between 0.0005 and 0.05 did not reach the threshold of significance, they were considered to provide suggestive evidence of a potential causal relationship.

## 3 RESULTS

### 3.1 Determination of IVs

Through the preset filtering criteria, IVs showing a causal association with circulating inflammatory proteins and BCC, SKCM, and cSCC were identified. The number of SNPs ranged from 18 to 46, with all *F*‐values greater than 10, indicating a strong correlation with the exposure factors (Table 1). Detailed information on the 476 SNPs (effect allele, standard error, palindromic sequence removal, etc.) is provided in Table S1.

**TABLE 1:** Instrumental variables of circulating inflammatory proteins associated with BCC, SKCM, and Cscc.

Outcome	Exposure	Reported trait	Data source	Sample size	Nsnp	Mean *F*
BCC	CCL4	C‐C motif chemokine 4	GWAS Catalog	14 744	31	72.1398
	CST5	Cystatin D	GWAS Catalog	14 736	46	69.3830
	EN‐RAGE	Protein S100‐A12	GWAS Catalog	14 743	23	28.7816
	FIt3L	Fms‐related tyrosine kinase 3 ligand	GWAS Catalog	14 734	43	36.4284
	IL‐1 alpha	Interleukin‐10	GWAS Catalog	14 744	32	27.3992
	TNFB	TNF‐beta	GWAS Catalog	11 792	37	102.4443
	TRANCE	TNF‐related activation‐induced cytokine	GWAS Catalog	14 736	43	36.1552
SKCM	CCL4	C‐C motif chemokine 4	GWAS Catalog	14 744	31	72.1398
	IL‐10	Interleukin‐10 receptor subunit alpha	GWAS Catalog	11 793	18	21.5413
	SCF	Stem cell factor	GWAS Catalog	14 736	42	37.9997
	Beta‐NGF	beta‐nerve growth factor	GWAS Catalog	14 743	35	22.7357
cSCC	CCL4	C‐C motif chemokine 4	GWAS Catalog	14 744	31	72.1398
	IL‐1 alpha	Interleukin‐10	GWAS Catalog	14 744	32	27.3992
	OSM	Oncostatin‐M	GWAS Catalog	14 736	22	27.2990

Nsnp denotes the number of single nucleotide polymorphisms (SNPs) utilized.

Abbreviations: BBC, basal cell carcinoma; Cscc, cutaneous squamous cell carcinoma; GWAS Catalog, genome‐wide association study; SKCM, cutaneous malignant melanoma.

### 3.2 Causal relationship between circulating inflammatory proteins and BCC, SKCM, and cSCC

Under the IVW method, evidence suggests causal effects exist for 11 circulating inflammatory factors on cutaneous‐origin exacerbated tumors. It was observed that variations in four inflammatory factors (CCL4, Flt3L, TNFB, and TRANCE) showed an inverse correlation with BCC. That is, as the expression levels of these factors decrease, the risk of BCC correspondingly increases. IL‐1 alpha exhibited the most significant positive regulatory effect on BCC (OR: 1.1768, 95% CI = 1.0666–1.2983, *p* = 0.0012). Additionally, an increase in IL‐10 abundance potentially mitigates the risk of developing SKCM (OR: 0.7772, 95% CI = 0.6483–0.9316, *p* = 0.0064), with CCL4 and SCF likely being positive factors for increased susceptibility to SKCM. Regarding cSCC, the study reveals positive promotional effects of IL‐1 alpha (OR: 1.2720, 95% CI = 1.0607–1.5254, *p* = 0.0094) and OSM (OR: 1.2001, 95% CI = 1.0235–1.4070, *p* = 0.0247), with a predicted increase in CCL4 levels associated with an 8.4% reduced risk (Figure 2).

**FIGURE 2:** Causal relationship between 11 circulating inflammatory proteins and BCC, SKCM, and cSCC (IVW method). BBC, basal cell carcinoma; Cscc, cutaneous squamous cell carcinoma; SKCM, cutaneous malignant melanoma.

Cochran's Q test excluded the presence of heterogeneity in the IVW method, and leave‐one‐out analysis revealed no SNPs significantly affecting the causal effect. Most importantly, there was no statistical significance in the MR‐Egger intercept test and MR‐PRESSO, indicating no interference from horizontal pleiotropy (Table 2).

**TABLE 2:** Initial causal association sensitivity tests of 11 circulating inflammatory proteins with BCC, SKCM, and Cscc.

		Cochran's Q		MR‐Egger intercept		MR‐PRESSO	
Outcome	Exposure	Q(IVW)	*p*	Egger‐intercept	*p*	Global *p*	Distort *p*
BCC	CCL4	23.4556	0.7960	0.0012	0.8100	0.734	NA
	CST5	50.0193	0.2808	−0.0009	0.7856	0.333	NA
	EN‐RAGE	21.2249	0.5069	0.0074	0.3250	0.494	NA
	FIt3L	61.3932	0.5269	−0.0013	0.7959	0.484	NA
	IL‐1 alpha	99.0794	4.817	−0.0014	0.9017	0.524	NA
	TNFB	37.4430	0.4027	−0.0066	0.1561	0.387	NA
	TRANCE	48.8074	0.2183	0.0122	0.1324	0.25	NA
SKCM	CCL4	39.4366	0.1162	0.0105	0.4327	0.166	NA
	IL‐10	20.1698	0.2656	−0.0113	0.5416	0.308	NA
	SCF	39.9053	0.5192	−0.0167	0.1171	0.505	NA
cSCC	Beta‐NGF	40.6441	0.2009	0.0270	0.1610	0.238	NA
	CCL4	29.5045	0.4912	−0.0014	0.9015	0.517	NA
	IL‐1 alpha	65.6590	0.2758	−0.0235	0.2642	0.484	NA
	OSM	14.9252	0.8267	−0.0181	0.2850	0.866	NA

Abbreviations: BBC, basal cell carcinoma; Cscc, cutaneous squamous cell carcinoma; IVW, inverse variance weighted; MR‐PRESSO, mendelian randomization pleiotropy residual sum and outlier; SKCM, cutaneous malignant melanoma.

### 3.3 Bayesian weighted MR validation

To further reinforce the robustness of the IVW method, this study employed BWMR to additionally validate the causal effects between circulating inflammatory proteins and cutaneous‐origin exacerbated tumors (Figure 3). Results confirmed that the direction of causal effects for all circulating inflammatory proteins and outcome factors was consistent. The *p*‐values for CST5 and EN‐RAGE related to BCC and CCL4 related to cSCC were all above 0.05, indicating these associations did not reach statistical significance. To avoid overinterpretation or misleading conclusions, nine inflammatory factors associated with cutaneous‐origin exacerbated tumors were ultimately identified.

**FIGURE 3:** Causal relationship between 11 circulating inflammatory proteins and BCC, SKCM, and cSCC (BWMR method). BBC, basal cell carcinoma; BWMR, Bayesian Weighted Mendelian Randomization; Cscc, cutaneous squamous cell carcinoma; SKCM, cutaneous malignant melanoma.

### 3.4 Causal relationships between BCC, SKCM, cSCC, and circulating inflammatory proteins

Using a threshold of *p* < 0.05, *kb = *10 000, *R* ^2^ = 0.001, and *F *> 10, 39–147 IVs related to cutaneous‐origin exacerbated tumors were identified and considered as exposure factors. On this basis, a reverse TSMR analysis was conducted in conjunction with circulating inflammatory proteins. The IVW method indicated that the causal effects between BCC, SKCM, cSCC, and the previously determined nine inflammatory factors were not significant and did not reach statistical significance (*p *> 0.05) (Figure 4).

**FIGURE 4:** Causal relationship of BCC, SKCM, and cSCC with nine circulating inflammatory proteins. BBC, basal cell carcinoma; Cscc, cutaneous squamous cell carcinoma; SKCM, cutaneous malignant melanoma.

### 3.5 Two‐step MR

To explore the mediating role of immune cell‐related traits as intermediary factors in the causal effects between circulating inflammatory proteins and BCC, SKCM, and cSCC, this study first identified 38, 39, and 35 immune cells with causal effects on BCC, SKCM, and cSCC, respectively, under the statistical threshold of *p* < 0.05 (Table S2). Subsequently, the study further estimated the causal relationships between the nine circulating inflammatory proteins, validated by the BWMR method, and 112 immune cell traits.

The analysis results indicate that, in BCC, IL‐1 alpha negatively regulates the proliferation of CD11b on CD14+ monocyte (OR: 0.7409, 95% CI = 0.5899−0.9305, *p* = 0.0099). Concurrently, the trend in Flt3L is consistent with two immune cells (CD4+ CD8dim T cell %lymphocyte and CD4+ CD8dim T cell %leukocyte). Regarding SKCM, 29 SNPs were selected as IVs for CCL4, based on which a negative correlation with three immune cell traits was identified. Notably, OSM significantly regulates three immune cells causally related to cSCC. Specifically, it is a positive factor for the growth of CD20 on IgD‐ CD38‐B cell (OR: 1.2342, 95% CI = 1.0369−1.4691, *p* = 0.0179) and CD4 on activated CD4 regulatory T cell (OR: 1.3947, 95% CI = 1.0115−1.9231, *p* = 0.0424), and is likely a potential disruptor for FSC‐A on granulocyte (OR: 0.7409, 95% CI = 0.5899−0.9305, *p* = 0.0099) (Figure 5). After Bonferroni correction, these causal relationships were not significantly associated (*p* < 0.0005). In sensitivity analyses, the removal of individual SNPs did not affect the causal effects between circulating inflammatory proteins and immune cells. The derived P values from Cochran's Q, MR‐Egger intercept test, and MR‐PRESSO were all greater than 0.05 (Tables [Link], [Link]), indicating no influence from heterogeneity or pleiotropy.

**FIGURE 5:** Causal relationship between 12 immune cell‐mediated circulating inflammatory proteins and dermal progression of tumors.

### 3.6 Calculation of potential mediating effects

To ensure the robustness of the mediating role of immune cells in the regulation of cutaneous‐origin exacerbated tumors by circulating inflammatory proteins, the selection of mediators was based on the significance of *p* values, integrating existing observational studies and clinical relevance. CD4+ CD8dim T cell %leukocyte, CD4‐CD8‐Natural Killer T %T cell, and CD20 on IgD‐ CD38‐B cell were ultimately chosen as mediating factors affecting the causal effect.

Through two‐step MR analysis, this study identified FIt3L as a potential protective factor for CD4+ CD8dim T cell %leukocyte (OR: 1.1894, 95% CI = 1.0359−1.3656, *p* = 0.0139), suggesting that the abundance of immune cells increases with the level of inflammatory factors. This viewpoint was further validated and expanded upon exploring the causal effects of CCL4 and OSM on immune cells. Additionally, a negative feedback regulatory mechanism of CD4+ CD8dim T cell %leukocyte on BCC was observed (OR: 0.9536, 95% CI = 0.9105−0.9987, *p = *0.0439). Conversely, the progression of SKCM is positively regulated by CD4‐CD8‐Natural Killer T %T cell (OR: 1.0762, 95% CI = 1.0016−1.1564, *p = *0.0450) and an increase in the expression level of CD20 on IgD‐CD38‐B cell raises the risk of cSCC by 9.2 percentage points (OR: 1.0921, 95% CI = 1.0093−1.1817, *p* = 0.0286) (Figure 6).

**FIGURE 6:** Causal relationship of circulating inflammatory protein‐immune cells‐BCC, SKCM, and Cscc. BBC, basal cell carcinoma; Cscc, cutaneous squamous cell carcinoma; SKCM, cutaneous malignant melanoma.

After determining the indirect effects, the mediating effects of the selected immune cells in the specific causal relationships were quantified using the product of coefficients method. Specifically, the mediating effect of CD4+ CD8dim T cell %leukocyte from FIt3L to BCC was ‐0.0082 (95% CI = ‐0.0323–0.0158), accounting for 9.26% of the total effect. In the causal relationship between CCL4 and CD4+ CD8dim T cell %leukocyte, the mediation percentage by CD4‐CD8‐Natural Killer T %T cell was 8.96%, with a mediating effect of 0.0078 (95% CI = ‐0.0201−0.0046). Additionally, CD20 on IgD‐CD38‐B cell mediated 10.16% of the causal effect between OSM and cSCC, with a mediating effect of 0.0185 (95% CI = ‐0.0188–0.0559) (Table 3).

**TABLE 3:** The proportion of mediated immune cells in the causal relationship between circulating inflammatory proteins and BCC, SKCM, and Cscc.

Outcome	Mediating factor	Total effect *β*all	Indirect effect *β*1	Indirect effect *β*2	Mediating effect	Mediating effect scale
BCC	CD4+ CD8dim T cell %leukocyte	−0.0891	0.1734	−0.0475	−0.0082	9.26%
SKCM	CD4‐CD8‐NaturalKiller T %T cell	−0.0870	−0.1062	0.0735	−0.0078	8.96%
cSCC	CD20 on IgD‐CD38‐B cell	0.1824	0.2104	0.0881	0.0185	10.16%

Abbreviations: BBC, basal cell carcinoma; Cscc, cutaneous squamous cell carcinoma; SKCM, cutaneous malignant melanoma.

## 4 DISCUSSION

Numerous observational studies have suggested a link between circulating inflammatory proteins and cutaneous‐origin exacerbated tumors.^19^, ^20^ However, potential confounding factors could introduce uncertainty in causal inference. To delve deeper into this relationship, based on extensive publicly available summary statistics, the TSMR method was used to identify potential causal effects of nine circulating inflammatory proteins on BCC, SKCM, and cSCC. Additionally, through two‐step MR analysis from a genetic perspective, three immune cells were determined to play significant regulatory roles in the causal effects of FLI3L, CCL4, and OSM on these three types of skin cancer, providing a solid theoretical basis for clinical decision‐making.

This study delved into the mediating pathways of specific immune cells in the causal relationships between circulating inflammatory proteins and common skin cancers. Specifically, CD4+ CD8dim T cell %leukocyte plays a negative regulatory role in the causal pathway where FIt3L inhibits the development and progression of BCC. Similarly, while confirming the adverse impact of CCL4 on SKCM risk, the mediating effect of CD4‐CD8‐Natural Killer T %T cell accounts for 8.96%. However, in the process where OSM promotes the risk of cSCC, CD20 on IgD‐CD38‐B cells demonstrates a positive role.

Proteomics, introduced by Marc Wilkins in 1994, plays a crucial role in cancer research and treatment as well as in the identification of malignant biomarkers.^21^ Inflammation, recognized as one of the hallmarks of cancer, has a dual role in the development and progression of tumors.^22^ This study focuses on circulating inflammatory proteins, exploring their potential mechanistic roles in specific skin cancers. Research on the anti‐tumor properties of Flt3L is not new. As early as 1998, Flt3L administration was proven to effectively inhibit the growth of murine SKCM and could potentially modulate immune therapy for cutaneous‐origin exacerbated tumors.^23^ Moreover, Liu et al.^24^ confirmed through a series of clinical trials that upregulating Flt3L expression could enhance immune responses and improve the efficacy of anti‐cervical cancer vaccines, revealing Flt3L's significant role in the pathological process of cervical cancer. This study delves into the genetic‐level exploration of Flt3L's inhibitory effects on BCC, yet robust research establishing their causal relationship is still lacking.

CCL4, located on the long arm of chromosome 17 at region 12, is also known as Macrophage Inflammatory Protein‐1α. As one of the 28 CC chemokines, it plays a critical role in regulating immune cell functions and modulating tumor progression and metastasis.^25^ A case–control study involving 314 Han Chinese patients with breast carcinoma (BC) and 209 healthy individuals identified CCL4 as a potential therapeutic target for BC.^26^ Building on experimental research, the team led by Shamoun et al.^27^ demonstrated that the expression level of CCL4 protein is associated with a 30% reduction in cancer survival rates in colorectal cancer patients. Huang et al.,^28^ through bioinformatics analysis and immunohistochemistry validation, determined that chemokines including CXCL9, CXCL10, and CCL4 play a positive role in enhancing the overall survival of patients with SKCM. This study, after limiting the impact of confounding factors, reached a consistent conclusion. Given the scarcity of clinical studies on CCL4 and SKCM, this finding can provide a basis for subsequent biological experiments.

OSM, a member of the interleukin‐6 family, is composed of 209 amino acid residues. It has been shown to exert inhibitory effects on colorectal cancer, chondrosarcoma, and glioblastoma, among others.^29^ However, inhibiting OSM has also emerged as a novel therapeutic strategy for various tumors. OSM leads to an increase in circulating tumor cells and a decrease in survival levels in breast cancer (BC), making it a potential cytokine that exacerbates cachexia in BC patients.^30^ In cervical cancer, OSM exacerbates the poor prognosis by inducing STAT3.^31^ Simonneau et al.^19^ initially identified the pro‐tumoral role of OSM in cSCC through mouse experiments. Moreover, OSM is significantly associated with other types of squamous cell carcinoma. In keratoacanthoma, a condition similar to cSCC, OSM has been proven to be highly expressed.^32^ Additionally, in a study examining the link between inflammatory biology and esophageal squamous cell carcinoma, OSM was also found to be associated with poorer prognoses.^33^ By reviewing existing epidemiological results, the study reaffirms the positive causal relationships between the identified sets of circulating inflammatory proteins and cutaneous‐origin exacerbated tumors, offering new insights into understanding and exploring the pathogenesis of skin cancers.

Research indicates that CD4‐CD8‐Natural Killer T cells also play a suppressive role in the causal effects of CCL4's negative regulation on SKCM. Indeed, upon successful activation, NKT cells secrete substances such as perforin and tumor necrosis factors, serving as a critical line of defense against external infections and malignancies. In clinical practice, NKT cell therapy is particularly suited for cancer patients who have developed resistance to long‐term medication.^34^ Ma et al.^35^ revealed through mouse experiments that controlling the growth of liver cancer can be achieved by regulating the levels of CXCL16 to influence NKT cell activity. Moreover, clinical trials and comparative analyses of tumor size before and after treatment in non‐small cell lung cancer and head and neck tumors further substantiate the negative impact of NKT cells on tumor progression.^36^ Although this study enhances our understanding of NKT cells' inhibitory role in tumor development, it is regrettable that definitive conclusions from double‐arm studies regarding their clinical efficacy remain elusive. Additionally, circulating inflammatory factors play a pivotal role in maintaining immune balance. It has been discovered that 24 h post‐administration of CCL4, there is a significant increase in the number of CD11b+ Kupffer cells in acute liver injury.^37^ Similarly, Amati et al.^38^ observed in lymphoma cell line biological experiments that CCL3, CCL4, and CCL5 inhibit the maturation and release of the pro‐inflammatory cytokine interleukin‐1β. These studies collectively unveil the complex regulatory mechanisms of CCL4 on immune cells.

Flt3L, also known as FLT3LG, is commonly associated with the FLT3 receptor, playing a crucial role in the regulation of hematopoietic cell proliferation and differentiation. A plethora of clinical studies suggest that Flt3L may exert an anti‐cancer effect by stimulating dendritic cells.^39^ Notably, Zhang et al.^40^ discovered in a BCG immunotherapy study for bladder cancer that FLT3LG enhances the ex vivo activation of CD8 T cells, providing a novel candidate target for future optimization of cancer treatments. This research delves into the critical role of Flt3L in regulating CD4+ CD8dim T cell percentage in leukocytes, unveiling the genetic mechanisms by which it inhibits the progression of BCC. However, robust clinical research establishing their causal relationship is still lacking. A previous TSMR study concerning immunophenotypes and type 2 diabetes revealed the stimulatory effect of the absolute count of CD4+ CD8dim T cells on outcome factors.^41^ Moreover, Parrot et al.^20^ found that the interleukin‐9 receptor enhances the immune function of double‐positive T cells in SKCM by protecting them from apoptosis. In summary, various circulating immunoproteins play a role in cancer promotion or suppression by regulating immune cells.

Contrary to normal cells, cancer stem cells possess the capability for self‐renewal and differentiation, serving as primary drivers for the onset, progression, and recurrence of tumors. As one of the key stem cells in SKCM, the proliferation of CD20+ cells results in a more pronounced formation of melanoma spheroid cells.^42^ In systemic non‐Hodgkin's lymphoma, selective radioimmunotherapy targeting CD20+ tumor cells has been proven effective.^43^ Building on this, our study preliminarily identifies the promotional role of CD20 on IgD‐CD38‐B cells in cSCC. Liu et al.^19^ have used bioinformatics tools to reveal that in cholangiocarcinoma, differentially expressed genes with high OSM expression are enriched in immune response‐related pathways. However, there is currently no definitive evidence to determine whether OSM levels positively stimulate or negatively inhibit CD20 expression.

From the current literature, this study is the first to investigate the mediating role of immune cells in the causal relationship between specific circulating inflammatory factors and the exacerbation of skin‐derived tumors. While revealing significant associations, several limitations must be acknowledged. First, the genetic summary data utilized in the study were exclusively derived from European ancestry, which, while reducing population‐specific confounding factors, limits the generalizability of the results to other ethnicities. Second, to obtain as many IVs as possible, within an acceptable range, the threshold for SNP selection was expanded to 1e‐5. Lastly, although MR tools are considered robust for exploring causal relationships, validation of results through biological control experiments is equally crucial.

In conclusion, this study delves into the causal relationships between circulating inflammatory proteins, immune cell phenotypes, and three types of skin‐originated exacerbating tumors. Employing a Two‐step MR approach, we successfully identified three sets of strong intermediary relationships and explored the mediating effects of immune cells. These findings hold promise for guiding the identification of potential biomarkers and therapeutic targets for BCC, SKCM, and cSCC.

## Supporting information

Supporting Information

Supporting Information

Supporting Information

Supporting Information

## Data Availability

The data that support the findings of this study are openly available in the GWAS Catalog at https://www.ebi.ac.uk/gwas/, reference number GCST90274758‐GCST90274848.
